The article "Melioidosis: Clinical impact and public health threat in the tropics" was retracted in 2020. Reasons: errors in the data; errors in the analysis; errors in the results or conclusions; errors in the text.

# Melioidosis: Clinical impact and public health threat in the tropics

**DOI:** 10.1371/journal.pntd.0004738

**Published:** 2017-05-11

**Authors:** Ramar Perumal Samy, Bradley G. Stiles, Gautam Sethi, Lina H. K. Lim

**Affiliations:** 1 Department of Physiology, NUS Immunology Programme, Centre for Life Sciences, Yong Loo Lin School of Medicine, National University Health System (NUHS), National University of Singapore, Singapore; 2 Integrated Toxicology Division, US Army Medical Research Institute of Infectious Diseases, Fort Detrick, Maryland, United States of America; 3 Department of Pharmacology, Yong Loo Lin School of Medicine, NUHS, National University of Singapore, Singapore; George Washington University, UNITED STATES

## Abstract

This review briefly summarizes the geographical distribution and clinical impact of melioidosis, especially in the tropics. *Burkholderia pseudomallei* (a gram-negative bacterium) is the major causative agent for melioidosis, which is prevalent in Singapore, Malaysia, Thailand, Vietnam, and Northern Australia. Melioidosis patients are increasingly being recognized in other parts of the world. The bacteria are intrinsically resistant to many antimicrobial agents, but prolonged treatment, especially with combinations of antibiotics, may be effective. Despite therapy, the overall case fatality rate of septicemia in melioidosis remains significantly high. Intracellular survival of the bacteria within macrophages may progress to chronic infections, and about 10% of patients suffer relapses. In the coming decades, melioidosis will increasingly afflict travelers throughout many global regions. Clinicians managing travelers returning from the subtropics or tropics with severe pneumonia or septicemia should consider acute melioidosis as a differential diagnosis. Patients with open skin wounds, diabetes, or chronic renal disease are at higher risk for melioidosis and should avoid direct contact with soil and standing water in endemic regions. Furthermore, there are fears that *B*. *pseudomallei* may be used as a biological weapon. Technological advancements in molecular diagnostics and antibiotic therapy are improving the disease outcomes in endemic areas throughout Asia. Research and development efforts on vaccine candidates against melioidosis are ongoing.

## Introduction

*B*. *pseudomallei* is the causal agent of melioidosis (in Greek, “melis” means “distemper,” “oid” means “resemblance,” and “osis” means “condition”) [1]. Captain Alfred Whitmore and his assistant isolated this bacterium from morphine injectors at the Rangoon General Hospital in Burma in 1911–1912. This bacterium originates in muddy water as well as humid soil and is prevalent in many tropical countries. Melioidosis has not only become a serious veterinary problem but can infrequently affect humans. A severe animal outbreak was first reported in Kuala Lumpur in 1913, and Singapore reported its first case in 1920. Later, Krishnaswami reported nearly 100 human cases in Rangoon [2]. Several sporadic human cases were reported after the Second World War [3]. The organism can be grown from clay soils, most commonly at a depth of 25–45 cm [4]. Ingestion is one of the most common ways for humans to contract melioidosis, and the infection is widely spread during the rainy season [5]. Although the worldwide distribution of infection is currently unclear, this review illustrates current information about the soil isolates, epidemiological investigations, global presence, and clinical impact of melioidosis upon human health.

The article "Melioidosis: Clinical impact and public health threat in the tropics" was retracted in 2020. Reasons: errors in the data; errors in the analysis; errors in the results or conclusions; errors in the text.

## Transmission and clinical features of melioidosis

Melioidosis mainly affects susceptible persons who are directly in contact with contaminated wet soils. Immunosuppressed elderly persons (e.g., those suffering from diabetes mellitus and/or alcoholism) are at increased risk of developing infection. *B*. *pseudomallei* is also responsible for fibrosis [6] and chronic lung diseases [7]. The disease spreads throughout endemic areas during the rainy season [8,9], but outbreaks are also well documented in dry areas due to contaminated water and soil [10]. Although melioidosis is mainly transmitted by inhalation, it may occasionally be acquired via nosocomial infections, laboratory accidents, vertical transmission at childbirth, and sexual contact [11,12]. The disease has protean manifestations ranging from localized abscess formation to disseminated abscesses, septicemia, shock [13–15], and possible death [15,16–20]. The lungs are the most common organ affected by this disease; affected lungs lead to abscesses and septicemic spread. Many patients become acutely septicemic, as reported in Malaysia, Singapore, Thailand, and Northern Australia [21]. However, central nervous system involvement in melioidosis is rare [22]. A number of septicemic patients have been also diagnosed with melioidosis [23]. Several localized and septicemic melioidosis outbreaks also occurred after a tsunami in 2004 [24–25]. A previous study showed that a Singapore Army soldier was also affected severely by cutaneous melioidosis [26–28].

## Geographical distribution, disease incidence, and ecology

This bacterium is relatively narrow in its worldwide distribution to the temperate regions with proven cases of melioidosis (Table 1) [29]. The areas of high endemicity, possible endemicity (higher number of cases reported recently), sporadic presence, environmental isolates only, and unconfirmed travel history/only serology evidence are indicated. Sporadic cases have also been reported in Pakistan, India, Bangladesh, Indonesia, Philippines, Sri Lanka, Papua New Guinea, Madagascar, France, Mexico, Brazil, Colombia, Venezuela, Ecuador, the Middle East (Iran), and the Caribbean (Fig 1). These bacteria are naturally found mainly in environmental water or moist soil, which includes rice fields, but they can also survive in tap water meant for human consumption [30].

The article "Melioidosis: Clinical impact and public health threat in the tropics" was retracted in 2020. Reasons: errors in the data; errors in the analysis; errors in the results or conclusions; errors in the text.

**Table 1:** Global distribution of melioidosis outbreak, incidence, and their reported cases (an overview).

Melioidosis outbreak (reported cases)					
Highly endemic areas with cases	Possible endemic areas; multiple cases, significant numbers of exported cases	Epidemic; limited outbreak	Sporadic case reports	Unconfirmed identification, uncertain travel history, or serological evidence only	Isolates from environment only
Burma (100) [206] Malaysia (406) [207] Singapore (372) [18,43] Thailand (800) [208] Vietnam (300) [78] Northern Australia (252) [168, 221]	Brunei (45) [37] Taiwan (40) [207] Cambodia (5) [38] Hong Kong (6) [78,209] Southern China (8 per year-) [210]	France [7]	Bangladesh (5) [82,211] India (95) [7] Indonesia (4) [212] Guam (2) [210] Japan (1) [213] Philippines (1) [214] Pakistan (10) [214] Sri Lanka (1–3) [81] Papua New Guinea (-) Iran (7) [38] Madagascar (1) France (3) Mexico (1) [152] Brazil (1) [38] Colombia (1) [38], Venezuela (1) [38] Ecuador (1) [38]	United States of America (5) United Kingdom (33–49) [38] Niger (0) South Africa (0) Kenya (0) Egypt (0) Spain (1) [38] Germany (1) [38] South Korea (2) [38] Turkey (49) [38] Saudi Arabia (4) [93] United Arab Emirates (2–7) [93]	Peru (1) [38] Italy (1) [215] Cote d’Ivoire (1) [38] Uganda (0) Haiti (1) [38] Reunion Island (1) [38]

-: unconfirmed travel cases.

**Fig 1:** Global geographical distribution of melioidosis. The areas of high endemicity in Southeast Asia (Thailand, Vietnam, Cambodia, Malaysia, and Singapore)/Northern Australia. Possible endemic, sporadic areas, environmental isolates only, and unconfirmed travel history/only serology evidence are indicated. However, sporadic cases have been reported throughout the world in Pakistan, India, Bangladesh, Indonesia, Philippines, Sri Lanka, Papua New Guinea, Madagascar, France, Mexico, Brazil, Colombia, Venezuela, Ecuador, the Middle East (Iran), and the Caribbean.

### Singapore

The prevalence of this infection is 0.2% among the population in Singapore, yet it is related to huge death and relapse rates. An earlier study showed that of 12 patients, 6 had relapsed and 2 died [31]. As just one example, a 43-year-old male suffered with persistent pain in the left thigh, high fever, and weight loss due to musculoskeletal melioidosis masquerading as diabetic amyotrophy. This disease is readily treatable but also represents a diagnostic challenge when it occurs at uncommon sites [32]. There was a total of 112 deaths, representing a fatality rate of 16.2%, during the period of 1998–2007 in Singapore [33], which is much higher than other countries like Thailand [34]. Recently, the apparent increase of melioidosis in Singapore has been partly attributed to increased social awareness and improved diagnostic techniques. However, another causative factor might be too much soil excavation generating aerosols and releasing the bacteria into the air [35]. Nearly 160 new cases were reported during 1995–1996 by occupational groups; over a quarter of those (26.9%) were cleaners, laborers, related workers, and drivers [36].

The article "Melioidosis: Clinical impact and public health threat in the tropics" was retracted in 2020. Reasons: errors in the data; errors in the analysis; errors in the results or conclusions; errors in the text.

### Thailand

The first case of melioidosis was reported in Thailand in 1955 [37], 3 indigenous cases were later reported in 1966 [38], and nearly 800 cases were reported in 1985 [24,39]. 602 patients with melioidosis were identified between 1986 and 1991. 42% of deaths were reported in the hospital [40]. Nearly 118 adult patients under went long-term treatment, among which 27 patients were culture-positive with relapses of melioidosis (3 patients relapsed twice), yielding a 15% relapse rate per year. The median time from discharge to relapse was 21 weeks (range of 1–290 days). The average time interval of hospital discharge to relapse was approximately 147 days (ranges of 1–290 days). Overall, 47% of septicemia patients had a relapsed disease, and 27% subsequently died. Severe septicemia patients were found to have clinical relapses 4.7 times (95% CI 1.6–14.1) greater than localized melioidosis patients [40]. Generally, the death rate was 21%, of which 39% were septicemic cases versus only 4% for nonsepticemic cases [25]. 89% of clinical cases were detected by culture of *B*. *pseudomallei*, while other cases were confirmed by an indirect hemagglutination antibody titer of 1:16 or greater [41,42].

### Vietnam

Melioidosis cases have been documented in soldiers stationed in various regions throughout Vietnam. Military personnel serving in Vietnam have been reported with acute and fatal melioidosis [43,44] (for example, they were diagnosed with septicemic melioidosis following acute influenza [45]). About 100 melioidosis cases were reported during the war of Vietnamese independence, during or after 1948–1954 [43,46]. More than 300 cases of melioidosis were subsequently diagnosed among American troops in Vietnam [47]. Some military dogs stationed in Vietnam were also infected by this bacterium, developing high fever, myalgia, and dermal abscesses. A remarkable number of melioidosis cases have also been reported among helicopter crews, which suggests that inhalation of either dust or aerosolized contaminated water can be another factor for exposure during dustoffs [43,48]. In addition, there is strong evidence of chronic infections among American troops due to exposure during time served in Vietnam, leading to fatal septicemia after the war and upon returning to the United States. A study estimated that roughly 225,000 Americans were potentially exposed to this bacterium while in Vietnam [49].

The article "Melioidosis: Clinical impact and public health threat in the tropics" was retracted in 2020. Reasons: errors in the data; errors in the analysis; errors in the results or conclusions; errors in the text.

Clinical surveillance and environmental sampling in southern Vietnam (1992–1998) showed only 9 *B*. *pseudomallei* infected cases (0.25%) among 3,653 blood cultures from febrile patients admitted to the Centre for Tropical Diseases in Ho Chi Minh City [50]. Soil samples were also collected from 407 sites in 147 paddy fields, including the 5 most important roads radiating from Ho Chi Minh City. *B*. *pseudomallei* was detected from 73 sites (18% of total sites tested); however, only 21% of the isolates were of the virulent L-arabinose (ara)-negative variety from 9 different rice fields. The low incidence of melioidosis in the provinces around Ho Chi Minh City can be attributed to the restricted distribution of *B*. *pseudomallei* in the soil throughout the area [51]. There were patients who also traveled in the Far East and developed pulmonary melioidosis first, further complicated by fatal encephalitis [52]. Pleuropulmonary melioidosis has also been reported in a Cambodian refugee who fled to Vietnam [53]. The first case of pulmonary melioidosis was reported in southern Cambodia. For example, a 58-year-old male patient and a 49-year-old female patient presented with respiratory illness and severe lung abscesses [54]. Subsequently, another 2 melioidosis cases were documented in Cambodian residents in Canada, as well as the United States. Both the patients had lived for several years in refugee camps in Thailand [53,55]. A more recent study analyzed the burden of melioidosis in Cambodia: out of 300 positive sputum samples, *B*. *pseudomallei* was isolated in 40%. Among patients who died during hospitalization, 32% were infected with *B*. *pseudomallei* [56,57].

### Australia

Melioidosis was first described in Australia (in North Queensland) following a 1949 outbreak in sheep [13]. A melioidosis patient with idiopathic pulmonary hemosiderosis was also reported in Central Australia [58]. A previous report suggested that 252 human cases of melioidosis were documented from 1990 to 2000 in Northern Australia. Of those, 46% were bacteremic and 19% died [7]. Nearly 50% of patients had pneumonia (15% with genitourinary infections and 18% with prostatic abscesses). Other clinical appearances included skin abscesses (13%), soft tissue abscesses (4%), osteomyelitis and/or septic arthritis (4%), and encephalomyelitis (4%). Several risk factors were associated with disease, such as diabetes (37%), extreme consumption of alcohol (39%), chronic lung disease (27%), renal disease (10%), and eating of kava (8%). The fatality rate was only 2% among patients without any risk factors [7].

The article "Melioidosis: Clinical impact and public health threat in the tropics" was retracted in 2020. Reasons: errors in the data; errors in the analysis; errors in the results or conclusions; errors in the text.

The spreading of melioidosis was mainly due to importation of animals from the temperate region of Northern Australia. *B*. *pseudomallei* isolates were collected from temperate areas in the Southwest and Western regions of Australia, and molecular typing reveals similar clonality for the past 25 years. Melioidosis is endemic throughout Northern Australia and Queensland, according to an epidemiology report on melioidosis from 2001 and 2002 [7]. The annual incidence was 5.8 cases per 100,000, whereas a higher incidence of 25.5 cases per 100,000 was noteworthy among native Australians. A significant number of melioidosis patients died from the disease, and overall, the total mortality rate was around 21%. Melioidosis-related morbidity and mortality remain quite high in native Australians, despite development of novel treatment modalities for managing this disease [59,60]. Previously, an Australian scientist reported that this bacterium can also be favorably grown from clay soils, typically at a depth of 25–45 cm [4].

### Taiwan

Melioidosis is an important disease in Taiwan. *B*. *pseudomallei* infection has been documented in a patient who acquired the infection by aspiration of river water in Philippines during a near-drowning incident [61]. Nearly 60% of the patients in Taiwan had primary infections, while 67% of patients were affected by secondary bacteremic pneumonia from 1982–2000. However, such infections were diagnosed only in 15 patients. Approximately 76% of infections (13 patients) were considered to be of native origin, among which 4 patients died of melioidosis, and 8 patients recovered from *B*. *pseudomallei* infection (1996–2000). One patient was a 56-year-old man working as a ranger at Ken-Ting Farm in southern Taiwan. He had been to Thailand for sightseeing 5 years before [62]. The patient’s blood cultures grew *B*. *pseudomallei* on the fifth day following admission. Another patient died by the ninth day, despite intensive care and a broad-spectrum antimicrobial regimen [63]. Melioidosis should be included in the reportable diseases, and its prevalence in Taiwan should be monitored, as comprehensive data are lacking.

The article "Melioidosis: Clinical impact and public health threat in the tropics" was retracted in 2020. Reasons: errors in the data; errors in the analysis; errors in the results or conclusions; errors in the text.

### India

Several cases have been reported from different regions of India, but only a few medical centers have successfully identified this bacterium [64–69]. For example, a noticeable epidemic of plaguelike illness was caused by *B*. *pseudomallei* [70,71–72], which was later clinically confirmed as melioidosis [64,66]. Chronic melioidosis has also been reported in cystic fibrosis patients of Indian origin [45]. In India, melioidosis has acquired the status of a newly upcoming transmittable disease [73]. A previous study of patients also revealed that skin/soft tissue (24%), liver abscesses (16%), and bones and joints (16%) were the important sites of this disease amongst those with diabetes. Moreover, septicemia and organ failure resulting in death were not uncommon [74].

### Other Asian countries

In other parts of Asia, infrequent cases of melioidosis from Indonesia were reported in the Dutch literature [75]. However, these diseases also constituted up to 10% of autopsy deaths in Rangoon, Burma in the year 1945. Only one case was reported in a Dutch traveler [76], with a second potential case in a Taiwanese traveler. A small number of locally acquired melioidosis cases have also been reported in Hong Kong [77–78]. However, a seroprevalence rate of 14% was confirmed by indirect hemagglutination assay in a tuberculosis sanatorium [79]. A few cases have also been identified in Sri Lanka [80]. Intermittent cases of melioidosis in travelers from Bangladesh have also been reported [7,81–82], together with 3 patients presenting septic arthritis after travel to Syhet [83]. Transmission was also documented in a 24-year-old Malaysian female patient who developed acute, nonfatal septicemic melioidosis after inhaling infective dust during a blast injury [84].

### Africa

Sporadic cases of melioidosis have been reported in Nigeria, Gambia, Kenya, and Uganda; however, the overall situation in Africa is uncertain [60,85–87]. Strikingly, only a few human cases have been previously reported in Africa. Wall et al. [88] reported a case in Gambia in a patient originally from Sierra Leone. Bremmelgaard et al. [89] noted a case in a Danish patient who had most likely acquired the infection in Kenya. Despite the paucity of clinical cases reported from Africa, serological surveys suggest that the causative organism is present in a number of countries, including Burkina Faso [90] and Uganda [91]. Additionally, *B*. *pseudomallei* has also been detected in the soil and animals in various African countries [92,93]. A recent report showed melioidosis associated with travel to Nigeria in a woman with diabetes, a major predisposing factor for this infection [86]. The first case of imported melioidosis was reported in Spain in a diabetic immigrant who visited West Africa during the rainy season [87].

The article "Melioidosis: Clinical impact and public health threat in the tropics" was retracted in 2020. Reasons: errors in the data; errors in the analysis; errors in the results or conclusions; errors in the text.

Infrequent cases of melioidosis have also been documented in other moist regions, such as Mauritius. The first case was reported in Madagascar in 1936 after isolation of *B*. *pseudomallei* in the lymph node of a pig [94]. Galimand and Dodin [95] previously isolated this bacterium in soil samples collected from the zoo of Antananarivo. However, no human case of melioidosis has been reported in Madagascar so far. An imported case of septicemic melioidosis occurred in a French expatriate living in East Madagascar [96], but not enough detail was available related to the travel history. Interestingly, this patient never traveled to prevalent regions and was never exposed to the infectious agent in France [97]. However, 6 years ago, the patient spent 1 week at a holiday resort in Mauritius during the dry season. Another study showed that an autochthonous case of melioidosis was acquired in Madagascar [98]. A recent case involving a young boy with laboratory-confirmed melioidosis has been reported from Malawi in 2011 [99].

### Latin America

Melioidosis patients with chronic granulomatous infection or diabetes have been reported during the rainy season in Puerto Rico [100–103]. Periodic cases of melioidosis were documented in Ecuador, Guadeloupe, Aruba, and Brazil [104]. Animal (sheep, goats, and pigs) outbreaks also occurred in Aruba during the 1950s [105], and the cause of infection was possibly a child with cystic fibrosis [106]. Previously, infrequent cases of melioidosis were also reported in Central and South America [107]. The first case of septicemic melioidosis was documented in northeastern Brazil in 2003 by culture of *B*. *pseudomallei* from a 10-year-old boy [108]. More recent cases have also been reported from a cluster in Ceara and other districts, further supporting Brazil as being endemic for melioidosis [109]. The various diverse suspected cases of septicemic melioidosis were recorded in another region within the state of Ceara, and a most striking example involves a woman who was washing clothes while sitting in a nearby river. She complained about a perianal abscess initially that persisted for 2 weeks before hospital admission with septicemia. After she died, *B*. *pseudomallei* was detected by blood culture [109]. There are published cases of nonbacteremic melioidosis in Colombia [110], Costa Rica, and Venezuela.

### United States of America

Glanders was eradicated from United States (US) domestic animals in the 1940s. However, a human case of glanders was documented in a Department of Defense laboratory worker (2000). Since 1945, this is the first human case of melioidosis infection reported in the US [111]. In addition, only a small number of isolated cases have been confirmed every year due to travelers, immigrants, and intravenous drug users [112]. The most intensely studied organism was the “Oklahoma isolates” from a soil-contaminated wound infection following a farming accident [113], which was identified as *B*. *pseudomallei* [114]. Later, the phylogenetic analysis placed these isolates in a separate group, apart from both *B*. *thailandensis* and *B*. *pseudomallei* [115,116].

The article "Melioidosis: Clinical impact and public health threat in the tropics" was retracted in 2020. Reasons: errors in the data; errors in the analysis; errors in the results or conclusions; errors in the text.

### Europe

Melioidosis is rare in Europe and is often linked with travel to Southeast Asia. The cases imported into the United Kingdom (UK) most likely occurred in immigrants from prevalent countries. Both human and animal cases have been imported from Bangladesh, Pakistan, India, Indonesia, and Philippines [117–120]. *B*. *pseudomallei* was isolated from 49 patients for the past decade. Almost 33 cases in the UK were diagnosed in patients after visits to Thailand, Bangladesh, and Australia, while 3 patients with cystic fibrosis also acquired the infection in Malaysia, the British Virgin Islands, or Brazil. Twenty-one clinical isolates of *B*. *pseudomallei* have been misidentified by European diagnostic laboratories during confirmation.

## Virulence and pathogenesis

*B*. *pseudomallei* possesses different types of secretion systems essential for its dissemination and intracellular survival [121]. The pathogenesis of melioidosis is partly attributed to exotoxins [122]. However, recent studies of the molecular and cellular basis of melioidosis pathogenesis show that *B*. *pseudomallei* is successfully transmitted from an environmental reservoir to lung epithelial cells via bacterial constituent-like capsules. The type III secretion system-3 (T3SS-3) activates and contributes to vacuolar escape and intracellular motility through BimA-mediated actin polymerization in infected epithelial cells [123–125]. In addition, the T3SS-3 plays an important role in evading killing by host autophagy. Activation of toll-like receptor-5 (TLR-5) by lipopolysaccharide (LPS) results in the rapid recruitment of innate immune cells, such as neutrophils, macrophages, and natural killer cells [126]. As a result, these cells release several proinflammatory cytokines, leading to associated host damage that provides an additional intracellular niche for bacterial replication. *B*. *pseudomallei* escapes by inducing cell-death (apoptosis), with secondary spread through the lymphatics and migrating macrophages containing the bacterium. The host often develops an adaptive immune response with T cells recruited in response to interferon-gamma (IFN-γ) production, which facilitates cell-mediated immune responses and antibody production after bacterial infection (Fig 2A and 2B) [127].

The article "Melioidosis: Clinical impact and public health threat in the tropics" was retracted in 2020. Reasons: errors in the data; errors in the analysis; errors in the results or conclusions; errors in the text.

**Fig 2:** Schematic representation showing the virulence and pathogenesis of melioidosis infection. *B*. *pseudomallei* is transmitted from its environmental reservoir to lung epithelial cells, where it initially attaches, possibly through bacterial components such as the capsule and type IV pili. Following invasion of epithelial cells, the T3SS-3 effectors assist in vacuolar escape and intracellular motility due to BimA-mediated actin polymerization. The activation of TLR-2, TLR-4, and TLR-5 by bacterial LPS and flagella results in recruitment of innate immune cells, such as neutrophils, macrophages, and natural killer cells. IRAK-M, interleukin-1-associated kinase 3; TLR, toll-like receptor; LPS, lipopolysaccharide; CD14, cluster of differentiation; NF-kB, nuclear factor kappa-light-chain-enhancer of activated B cells; IL, interleukin; TNF-α, tumor necrosis factor alpha; NLRC-4, NRL family CARD domain-containing protein 4; NLRP3, NACHT, LRR, and PYD domain-containing protein 3; ACS, acetyl-CoA synthetases; PCR, polymerase chain reaction.

Several animal models for studying *B*. *pseudomallei* pathogenesis have been investigated, including mice and nonhuman primates by intravenous (IV), intraperitoneal (IP), oral, subcutaneous (SC) and inhalation routes of infection [128–130]. This facultative intracellular pathogen contains a huge genome, which encodes a variety of virulence elements that promote survival in animal models by manipulating the host cell process and captivating elements of the host immune system. Various virulence factors play a vital role in *B*. *pseudomallei* infection, and these include capsular polysaccharide, LPS, adhesins, specialized secretion systems (i.e., typesII/IV and VI), actin-based motility, and myriad secreted factors that enable survival within a host and contribute to the pathogenesis of melioidosis [131,132]. For example, a recent study demonstrated that BALB/c mice exposed to mutant strains in an aerosol model using a lethal dose of *B*. *mallei* survived for 21 days versus mice exposed to wild-type bacteria that died within 4 days. Pathogenesis included modulating the host ubiquitination pathways, phagosomal killing, and actin–cytoskeleton rearrangement. Furthermore, virulence factors were associated with a host protein (BMAAO728) responsible for the closure of phagosomal membranes. The GABA(A) receptor-associated protein-like I, which is found in mice and humans and is responsible for cellular internalization, escape, evasion, and interaction with host proteins, involves BMAAO728 and BMAA1865/BMAA0553 [133]. There was a cluster of up-regulated genes, with one (BPSL1775) related to iron uptake receptor and pyocheline (pch/fptA) during lung infection in mice [134].

The article "Melioidosis: Clinical impact and public health threat in the tropics" was retracted in 2020. Reasons: errors in the data; errors in the analysis; errors in the results or conclusions; errors in the text.

Mice are extremely susceptible to acute respiratory infection caused by *B*. *pseudomallei*. Severe pathological symptoms of acute inflammation and necrosis are found in the lungs, liver, and spleen [135]. The murine model also reveals that diabetes increases the susceptibility to melioidosis [136]. *B*. *pseudomallei* (3 x 10^5^ CFU) was administered by different routes, such as IV, IP, SC, intranasal and orally, in mice, and the severity of infection and pathogenesis was compared. Bacterial loads were measured in various organs—such as the spleen, liver, lungs, lymph nodes, and brain—and blood after 3 days of infection. Bacterial loads did not show any tropism towards lung tissues after intranasal infection by a lethal dose of a highly virulent strain (NCTC 13178). However, the number of bacteria increased in the liver and spleen, but not in the lungs, of C57BL/6 and BALB/c mice after 24 h. Results clearly show systemic spread of *B*. *pseudomallei* from the lungs to other organs [137]. However, the mice infected by the IV or IP route demonstrated increased bacterial numbers (>10^6^ CFU) after day 2 of infection as a result of innate immunity not controlling infection that ultimately leads to sepsis and death. Pathogenesis caused by *B*. *pseudomallei* was studied by infecting mouse macrophages via intraperitoneal injection. Microscopic examination of U-937 macrophages infected with *B*. *pseudomallei* proves the occurrence of intracellular bacteria within membrane-bound vacuoles. In vitro study clearly shows that *B*. *pseudomallei* can survive and multiply in human phagocytes (Fig 3A and 3B). *B*. *pseudomallei*-infected mice have significantly large, confluent abscesses in the spleen (Fig 3D and 3E).

**Fig 3:** Ultrastructural examination of *B*. *pseudomallei* used for infection. (A) Scanning electron microscopy (SEM) image showing Bp before the infection with U-937 cells. (B) Bp-infected cells were examined by a transmission electron microscopy (TEM) with large number of bacilli (Bp) presented in the cytoplasm. Light micrograph showing *B*. *pseudomallei* infection of mouse spleen; section stained by Haematoxylin and Eosin (H&E) imaged with different magnification. (C–D) Large abscesses (Abs) with focal areas of necrosis, surrounded by a rim of meshed fibrous tissue (f) are evident after 2 weeks IP challenge with 1.7x105 CFU/ml. The bacterial invasion is more in spleen and liver than kidney. Bp, *B*. *pseudomallei*; abs, abscess; f, fibrous tissue; rs, rough surface; s, septa; sb, single bacilli; n, nucleus; ph, phagocytosis.

The article "Melioidosis: Clinical impact and public health threat in the tropics" was retracted in 2020. Reasons: errors in the data; errors in the analysis; errors in the results or conclusions; errors in the text.

Collectively, this mouse model may provide excellent data to better understand acute and chronic melioidosis in humans. Furthermore, these murine models of infection are similar to the acute and chronic disease in humans [138]. Earlier, studies also show that the type VI secretion system (T6SS-1) is important for virulence in a hamster model and can be positively regulated by the VirAG component system. T6SS-1 genes were overexpressed after internalization of these bacteria into the phagocytic cells, which leads to the formation of multinucleated giant cells in an infected monolayer [139,140].

The development of drug resistance by *B*. *pseudomallei* towards lysosomal defensins, cationic peptides, and cytotoxic lipids is quite remarkable [141]. The cell wall of this gram-negative bacterium naturally consists of LPS that harbors highly conserved, immunodominant antigens. Interestingly, high concentrations of antibodies against LPS2 are linked to decreased disease severity [142]. The pathogenic mechanism linked to endotoxin involves systemic effects on the mammalian host. Some of the bacteria-free filtrates of *B*. *pseudomallei* are lethal to mice, and elevated levels of endotoxin are released by mucin in the growth medium. Toxins present in culture filtrates can be precipitated by antisera. These toxic substances play an important role in the hemorrhagic (as well as necrotic) lesions and have been related to protease activity. The proteolytic enzymes, as well as a unique lethal exotoxin, are separable entities [143]. Furthermore, other polypeptides extracted from certain *B*. *pseudomallei* strains induce severe mortality after IP injection in mice [144]. The toxins produced by virulent, as well as avirulent, strains of *B*. *pseudomallei* are toxic to both hamsters and mice models. *B*. *pseudomallei* is generally able to survive within various cell lines and the process of phagocytosis, as examined from pathological sections. *B*. *pseudomallei* have several T3SS-3 that play important roles in bacterial survival and dissemination [145]. IFN-γ is important for innate immunity in animals [146]. Septicemic melioidosis is also associated with higher levels of cytokines that include tumor necrosis factor (TNF), interleukin-6 (IL-6), IL-10, IL-18, and IFN-γ. The TNF promoter polymorphism (TNF2 allele) is responsible for the severity of melioidosis. Utaisincharoen et al. [147] reported that mouse macrophages can easily invade *B*. *pseudomallei* in the absence of nitric oxide synthase (iNOS) production. This enzyme is essential for controlling the multiplication and survival of *B*. *pseudomallei* inside cells. In addition, IFN-γ and IFN-β (a type I interferon) are responsible for initiation of innate immunity against various microbial infections [148].

The article "Melioidosis: Clinical impact and public health threat in the tropics" was retracted in 2020. Reasons: errors in the data; errors in the analysis; errors in the results or conclusions; errors in the text.

### Cytokine responses and control of intracellular bacteria

Various studies clearly demonstrate that almost 50% of melioidosis patients have varying degrees of diabetes mellitus. Additionally, *B*. *pseudomallei*-infected diabetics have impaired IL-12P70 production that results in decrement of IFN-γ [149]. IL-12 assembly is poorly interconnected with lack of reduced glutathione (GSH) levels in diabetic patients. Adding GSH or N-acetylcysteine (NAC) to peripheral blood mononuclear cells in vitro specifically restores IL-12- and IFN-γ-induced clearing effects. Lack of GSH in mice increases susceptibility to melioidosis, and reduction of IL-12P70 leads to a poor outcome [150]. The close association between GSH impairment, diabetes, and augmented susceptibility to melioidosis can lead to a novel therapeutic option to control intracellular bacterial pathogens, especially in diabetic patients [151]. However, the immunocompromised ability of innate immune cells infected with *B*. *pseudomallei* to produce IL-12 and, subsequently, IFN-γ in response to certain infections hampers initiation of a proinflammatory response. IFN-γ is essential for inducing phagocytosis (e.g., by monocytes) and switching on potent bactericidal effects. A number of reports show that depleted GSH in antigen-presenting cells (APCs) can change T cell maturation into Th2 response. GSH or NAC addition of APCs results in a high level of IL-12 expression through a Th1 response [152–153].

## Laboratory diagnosis

Melioidosis is usually diagnosed by isolation and identification of *B*. *pseudomallei* from the sputum, urine, tissues, blood samples, and wound exudates. However, blood cultures have been confirmed negative just before death in the septicemic form of infection. This bacterium presents itself as a wrinkled colony on Ashdown’s selective agar (ASA) [154], whereas smooth colonies are produced on horse blood agar (HBA) or MacConkey’s agar [155,156]. The bacteria are gram-negative coccobacilli, with bipolar staining as observed in young cultures. Wrinkling of colonies is key to differentiation between *B*. *cepacia* (an opportunistic environmental pathogen) and *B*. *pseudomallei*; thus, further confirmatory tests, such as polymerase chain reaction (PCR), may be needed. Detection of bacteria-specific antibodies from a blood sample is another form of diagnosis. Serological tests revealing high-antibody titers are very useful in the presence of clinical diagnosis. Clinical diagnostic tests include agglutination, indirect hemagglutination, complement fixation, immunofluorescence, and enzyme immunoassays [156–158]. Cross-reactivity occurs in serological tests against *B*. *mallei*, which is recognized as a causative agent of glanders. Mainly, a direct immunofluorescent antibody test (DIF) is available for the quick diagnosis of melioidosis from patient sputum, pus, and urine. The DIF is more sensitive (73%) and of higher specificity (99%) versus culture of the bacterium from patients (*n* = 272) with a suspected case of melioidosis [159]. Furthermore, tests for pathogen-specific IgM and IgG are now commercially available for the confirmation of clinically suspected melioidosis. This is accomplished by using sera from bacteriologically confirmed melioidosis in high-risk patients. The sensitivities were, respectively, 100% for the IgG and 93% for IgM assays, while specificity was 95% for both assays [157, 160–162].

The article "Melioidosis: Clinical impact and public health threat in the tropics" was retracted in 2020. Reasons: errors in the data; errors in the analysis; errors in the results or conclusions; errors in the text.

## Antibiotic resistance and susceptibility/treatment of melioidosis

*B*. *pseudomallei* often develops resistance to existing antibiotics [163]. However, there is varying susceptibility to the various antibiotics, such as chloramphenicol, tetracyclines, trimethoprim-sulfamethoxazole, ureidopenicillins, cephalosporins, and clavulanic acid [164]. The second important cohort of antibiotics (cephalosporins, macrolides, rifamycins, colistin, and aminoglycosides) are not effective against *B*. *pseudomallei*. Third-generation antibiotics, including cephalosporins, are not clinically useful in treating melioidosis; however, carbapenems and amoxicillin-clavulanate are used for treatment with broad spectrum effects. Recently, combined therapy with trimethoprim and sulphonamides was noted to decrease bacterial growth [165]. Moreover, a treatment that combines chloramphenicol, doxycycline, and trimethoprim-sulfamethoxazole better controls the bacterium compared with individual treatment [165]. Fluoroquinolones have shown only weak activity during clinical trials against *B*. *pseudomallei* [166], but experimental evidence showed that it may be beneficial for immediate therapy or prophylaxis. *B*. *pseudomallei* develops resistance mechanisms against existing antibiotics due to enzymatic inactivation, target deletion, and efflux from the bacterium caused by chromosomally encoded genes. As a result, excessive production and mutations of the class A PenA β-lactamase can cause resistance to ceftazidime and amoxicillin-clavulanic acid. Deletion of the penicillin-binding protein-3 (PBP-3) leads to drug resistance towards ceftazidime. Similarly, over expression of the BpeEF-OprC drug-efflux pump causes resistance to trimethoprim (TMP) and TMP-sulfamethoxazole (SFZ) antibiotics [167] (Fig 4).

The article "Melioidosis: Clinical impact and public health threat in the tropics" was retracted in 2020. Reasons: errors in the data; errors in the analysis; errors in the results or conclusions; errors in the text.

**Fig 4:** Schematic diagram for melioidosis diagnosis and list of sensitive and resistance antibiotics. There are several factors, such as inactivation of enzyme, target deletion, and drug efflux pumps from the cells mediated by chromosomally encoded genes. Furthermore, the overproduction and point mutations in class A PenA β-lactamase affect some of the important drugs (i.e., ceftazidime and amoxicillin-clavulanic acid) that are responsible for the development of resistance mechanisms. However, the deletion of penicillin binding protein-3 (PBP-3) leads to ceftazidime resistance, and BpeEF-OprC efflux pump overexpression causes doxycycline, trimethoprim, and trimethoprim (TMP)-sulfamethoxazole (SFZ) resistance.

### Antibiotic synergism

In vitro screening assays have been established for the categorization of cytokines and antimicrobial drugs exerting synergistic activity for preventing intracellular pathogenesis of *B*. *pseudomallei*. IFN-γ was recognized as a potent antibacterial force against *B*. *pseudomallei* in infected macrophages by using this assay system. Third-generation cephalosporins combined with penicillin and aminoglycosides exert powerful effects [168]. Additionally, mice infected with a lethal dose of *B*. *pseudomallei* and then treated with subtherapeutic concentrations of ceftazidime and liposome-DNA-immune stimulatory complexes experience enhanced survival and completely clear the bacterial load compared to treatment with either therapeutic agent alone [168]. Therefore, immunotherapy can significantly enhance the efficiency of conventional antimicrobial treatment for melioidosis. However, lower doses of antibiotics are essential for the successful management and can also play an important role in eliminating remaining bacteria in a short-term treatment course [169]. In addition, the combination of antibiotic treatments has different courses of action on bacterial death. The combination of antibiotic treatment regimens not only strongly controls bacteria but also leads to significant synergistic effects [170–173]. The synergistic effect of aminoglycosides and β-lactams could be due to β-lactam damage of the cell wall that leads to increased intake of aminoglycosides [174]. It is very exciting to distinguish whether there is an observed synergism between these two antibiotics found to stimulate the envelope stress response after treatment. Furthermore, the complex-system-based quantitative methods are important for studying antibiotic relationships that also enable characterization of the molecular mechanism(s) of action, as well as affected cellular targets.

The article "Melioidosis: Clinical impact and public health threat in the tropics" was retracted in 2020. Reasons: errors in the data; errors in the analysis; errors in the results or conclusions; errors in the text.

The susceptibility of *B*. *pseudomallei* to antimicrobial agents has also been scrutinized [175–176] and, consequently, the treatment for melioidosis reasonably well established [27]. *B*. *pseudomallei* are variably susceptible to coamoxiclav but resistant to gentamicin and colistin. However, most melioidosis cases can easily be treated with suitable therapies. Early treatment must be initiated immediately after clinical diagnosis. Patients with acute melioidosis may die within hours or days unless prompt treatment is initiated. Long-term treatments with antibiotic combinations are needed for a complete cure. Although bloodstream infections with melioidosis are fatal, other forms of infection are usually nonfatal. Antibiotic therapies for the treatment of acute septicemic melioidosis have varying degrees of effectiveness.

*B*. *pseudomallei* is commonly susceptible to the following antibiotics: imipenem, penicillin, amoxycillin-clavulanic acid, azlocillin, ceftazidime, ticarcillin-vulanic acid, ceftriaxone, and aztreonam [23]. Based on randomized and semirandomized controlled clinical trials of drug regimens, effective treatments for severe acute human infection include intravenous administration of ceftazidime (with or without trimethoprim-sulfamethoxazole), amoxicillin-clavulanic acid, imipenem, and cefoperazone-sulbactam [36]. Meropenem is also used successfully to control the pathogen [177]. Oral treatment consists of chloramphenicol, trimethoprim-sulfamethoxazole, and doxycycline, although amoxicillin-clavulanic acid is also used alone or in combination therapy for acute infection. Doxycycline can be used to treat localized melioidosis, whereas combination with other antibiotics is required to alleviate systemic disease [21]. Thus, ceftazidime can be an important therapeutic option treatment along with other antibiotics such as cotrimoxazole or doxycycline (Table 2). Ceftazidime or meropenem are the therapeutic choice for treating severe cases of infection and can be given by the IV route for several weeks, followed by oral treatment (up to 20 weeks) with trimethoprim-sulphamethoxazole and doxycycline [178]. Mortality following septicemia and, presumably, adequate treatment is still 40%, whereas surviving patients may have a high relapse rate (4%–20%). Melioidosis can become chronic with formation of abscesses or remain subclinical for many years, probably since the microorganisms can survive within phagocytes with the risk of reactivation precipitated by immunosuppression. Pulmonary resection of abscesses is possibly essential for persistent cases of infection. The optimal treatment for chronic infections consists of intravenous ceftazidime for at least 2 weeks, followed by oral therapeutics given up to 3 months for the complete abolition of infection [179].

The article "Melioidosis: Clinical impact and public health threat in the tropics" was retracted in 2020. Reasons: errors in the data; errors in the analysis; errors in the results or conclusions; errors in the text.

**Table 2:** Randomized trials of potential antibiotic treatment in severe melioidosis. Recommendations for diagnosis, treatment and continuing care of melioidosis based on recent experience and best practice. Antibioti*c* treatment for severe infection is either intravenous Ceftazidime or Meropenem for several weeks, followed by up to 20 weeks oral treatment with a combination of trimethoprim-sulphamethoxazole and doxycycline.

Drugs	Enrolled	Number of patients		Duration days	Treatment failure	Mortality	References
		Melioidosis	Antibiotic dose				
Ceftazidime vs chloramphenicol+doxycycline+TMP/SMX	161	34 31	120 mg/kg/day 100 mg/kg/day	>7 4	0	37% 74%	[28]
Ceftazidime+TMP/SMX vs chloramphenicol+doxycycline+TMP/SMX	136	27 34	100 mg/kg/day 8+40 mg/kg/day 100 4+ 8+40	10–14	0	18.5% 47%	[216]
Ceftazidime vs amoxicillin-clavulanate	379	106 106	120 mg/kg/day 160	>7	39% 51%	47% 47%	[217]
Ceftazidime vs imipenem	296	106 108	120 mg/kg/day 50	>10	41% 20%	38% 36%	[218]
Ceftazidime Imipenem	34 34	68	100 mg/kg/day 50 mg/kg/day	2 g every 8 h 1 g every 8 h	20% 50%	35% 35%	[219]
Chloramphenicol+ trimethoprim-sulfamethoxazole+doxycycline	116	109	-	12 weeks	18.2% 46.5%	0	[180]
Ceftazidime amoxicillin/clavulanate	379	212 (56%)	120 mg/kg/day 160 mg/kg/day	-	0	47%	[217]
Ceftazidime co-trimoxazole trimethoprim, sulfamethoxazole, Chloramphenicol; doxycycline, trimethoprim, sulfamethoxazole,	73	64	100 mg/kg/day 8 mg/kg/day 100 mg/kg/day 4 mg/kg/day 8 mg/kg/d ay 40 mg/kg/day	3–6 months 10 14	0	18.5% 25% 30.7%	[216]
Cefoperazone/sulbactam + co-trimoxazole (vs ceftazidime + co-trimoxazole (trimethoprim)	84	20	25 mg/kg/day 8 mg/kg/day 100 mg/kg/day 8 mg/kg/day	-	0	0	[220]

Treatment failure is indicated by zeros (0).

Fluoroquinolones are given for treatment of acute melioidosis; however, this drug is not strongly recommended due to a high relapse rate. In addition, an in vitro study also clearly demonstrated that the minimum inhibitory concentrations (MICs) for some *B*. *pseudomallei* strains often exceed levels achieved in serum [180]. Ciprofloxacin (20 mg/kg/day) is administered individually or in combination with doxycycline for the management of melioidosis, despite some controversy as to whether ciprofloxacin can really penetrate through phagocytic cells where *B*. *pseudomallei* resides [179–181]. Ciprofloxacin serum levels of 2–3 mg/L have been achieved by standard oral dosage; hypothetically, intracellular doses of up to 20 mg/L can be achieved in macrophages. Additionally, serum levels of 9 mg/L are attainable by intravenous infusion, albeit for short periods [182].

The article "Melioidosis: Clinical impact and public health threat in the tropics" was retracted in 2020. Reasons: errors in the data; errors in the analysis; errors in the results or conclusions; errors in the text.

## Development of antibodies and vaccines for prevention of melioidosis

Several earlier reports have demonstrated that different types of genetically modified bacterial vaccines were evaluated to analyze their protective effects [183–185]. In addition, possible melioidosis vaccines, such as live attenuated, killed whole cell, dendritic cell (DC), and sub-unit plasmid DNA have been investigated for the prevention of disease [186].

The accessibility of several *B*. *pseudomallei* genome sequences has greatly aided the progress of vaccine target discovery for the alternative therapeutic and prophylactic strategies [187]. For example, researchers have discovered a very potent toxin known as *Burkholderia* lethal factor-1 (BLF-1) that prevents cells from breaking down protein in an infected host. Another study clearly demonstrated the potential of various DNA molecules from *B*. *pseudomallei* with vaccine potential [188].

There are two surface-associated antigens, capsular polysaccharide (CPS) and LPS, which are responsible for *B*. *pseudomallei* pathogenesis. Furthermore, two suitable monoclonal antibodies (mAbs) have been established that target the CPS and LPS to date [189]. The CPS mAb has been used for the identification of antigen from serum and urine of melioidosis patients. CPS individually, or in combination with an LPS mAb, prevents *B*. *pseudomallei* infection in mice. Although both mAbs confer protection when given singly, the combination treatment provided significantly better protection at low doses [189].

Until now, vaccines have not been developed commercially for the prevention of human melioidosis. Several novel vaccines for melioidosis are currently under development and being tested in animals [190–192]. However, well-established infection models are important for developing vaccines to assess efficacy and safety before human trials. The most effective immunity against melioidosis has been successfully obtained by using bacteria deficient in *ilvL*, *serC*, *aroB*, *purN*, *purM*, BPSS1509, *lipB*, *pabB*, *aroC* and *bipD* in *B*. *pseudomallei* vaccines [193,194]; subunit vaccines consisting of recombinant proteins (Hcp1, Hcp 2, Hcp 3, Hcp, LPS, Omp85), nonmembrane proteins (Lo1C, PotF, OppA), and outer membrane vesicles [139,195]; and components of the T3SS system (bipB bipC, bipD) [196]. For instance, a vaccination strategy containing a variety of components such as type VI secreted structural protein (recombinant *B*. *mallei* Hcp1), autotransporter protein (BimA), or type III secreted protein (BopA) and ABC transporter protein (*B*. *pseudomallei* Lo1C) reveals that BopA shows the greatest protection (60%–100% efficacy) against *B*. *mallei*- and *B*. *pseudomallei*-infected mice. Furthermore, serum obtained from the BopA-immunized mice was reactive with type III secreted bacterial recombinant proteins. T cells from vaccinated mice also show increased levels of IFN-γ [197,198].

The article "Melioidosis: Clinical impact and public health threat in the tropics" was retracted in 2020. Reasons: errors in the data; errors in the analysis; errors in the results or conclusions; errors in the text.

Additionally, an attenuated *B*. *pseudomallei bipD* mutant with dysfunctional T3SS-3 was employed to vaccinate mice. Incomplete defense was obtained in vaccinated mice after challenge with virulent wild-type *B*. *pseudomallei*, but inoculation with the purified *bip D* protein was not protective [199–200]. Attenuated whole-cell vaccines are not more protective than purified proteins against extracellular bacteria versus intracellular bacteria. The protective immunity induced by purified protein antigens is generally weaker due to non-cell-mediated immunity (CMI), which is important for abolition of antigens during the inactivation process [200]. With plasmid DNA vaccination, the antigen is expressed by the host cell and delivered directly to APCs, resulting in strong CMI [201]. A significant potential advantage of DNA vaccines is the ability to induce CD8^+^ T cell responses via MHC class I presentation, which is important for protection against intracellular pathogens [202]. In recent years, the focus of new vaccine development has largely been directed toward the use of discrete bacterial components known as subunit vaccines.

Moreover, previous human studies have demonstrated that the properties of oligopeptide-binding protein A (OppA Bp) may play a vital role in the ATP-binding cassette (ABC) transport system, because they can react with convalescent patient sera [203]. Recently, structural and computational approaches were also used to identify potential epitopes on OppA from *B*. *pseudomallei*. Synthetic peptides of this antigen were recognized by melioidosis patient sera [204,205]. This type of protein might be a potential target for developing vaccines and diagnostics against bacterial infections [190]. Therefore, several diverse strategies are essential for developing new vaccines against melioidosis.

### Future perspectives

Melioidosis continues to pose a potential threat, especially in Southeast Asian countries [168]. However, compared to several decades ago, current morbidity and mortality rates of melioidosis have significantly decreased due to better clinical management and advances in diagnostic techniques. Nonetheless, there remain many problems in the clinical management of this disease. The majority of younger patients develop acute pulmonary infection that often leads to multiple abscess formation with very high mortality rates. Therefore, melioidosis and its related diseases continue to directly or indirectly negatively impact the productivity and socioeconomic status of affected young adults in endemic countries. Low-cost, practical, accurate, and fast detection kits are not available in the market now. Until now, diagnosis has been mainly dependent upon bacterial growth in the laboratory. However, novel molecular methods of diagnosis (e.g., PCR) are being increasingly implemented for routine diagnosis. Despite the introduction of treatments based on intravenous administration of ceftazidime and carbapenem, the bacterium is still linked with high mortality and severe complications. For example, meropenem (25 mg/kg every 8 hours intravenously for ≥14 days) may be prescribed as an alternative treatment course for severe melioidosis [177,187]. Combination treatments are associated with side effects and lack of compliance, which are important considerations for patients requiring long-term oral drug treatment (e.g., given every 12 hours for up to several weeks). A long course of maintenance therapy with oral antibiotics is necessary to reduce the risk of relapse. Several vaccine strategies are currently being explored, but financial deficits may make immunization an impractical choice in several prevalent areas.

The article "Melioidosis: Clinical impact and public health threat in the tropics" was retracted in 2020. Reasons: errors in the data; errors in the analysis; errors in the results or conclusions; errors in the text.

Diabetes, open wounds, lung disease, and immune deficiency are important factors for melioidosis, and patients with those conditions must avoid direct exposure of contaminated clay soil and standing water in prevalent areas. In particular, persons engaged in agricultural activities (i.e., rubber plantation and paddy field work) must wear boots that can prevent direct infection via the feet and lower limbs. Standard precautions include wearing masks, gloves, and gowns to prevent infection, especially among healthcare workers attending to patients with melioidosis. In addition, clinicians examining travelers with severe pneumonia or septicemia returning from the subtropics or tropics should consider the differential diagnosis of acute melioidosis. Currently, *B*. *pseudomallei* vaccine candidates are not available for the prevention of melioidosis. After exposure to the causative organism, combination treatment with co-trimoxazole and doxycycline is recommended. Trovafloxacin and grepafloxacin are effective in animal models. In conclusion, more work and research remains to be carried out to better manage and prevent *B*. *pseudomallei*-related diseases that afflict not only humans but also animals.

**Key learning points**

- *Burkholderia pseudomallei* is the causative agent of melioidosis, which is prevalent throughout Southeast Asia.
- This bacterium is an important bioweapon and bioterrorism risk worldwide.
- The overall fatality rate of septicemia in melioidosis is very high, and bacteria are intrinsically resistant to many antimicrobial agents.
- Melioidosis increasingly affects travelers visiting endemic areas, thereby leading to septicemia.
- Clinicians should consider acute melioidosis as a differential diagnosis.

The article "Melioidosis: Clinical impact and public health threat in the tropics" was retracted in 2020. Reasons: errors in the data; errors in the analysis; errors in the results or conclusions; errors in the text.

**Top five papers**

1. Limmathurotsakul D, Kanoksil M, Wuthiekanun V, Kitphati R, deStavola B, Day NPJ, Sharon J. Peacock SJ. Activities of daily living associated with acquisition of melioidosis in Northeast Thailand: A matched case-control study. *PLoS Negl Trop Dis* 2013; **7**: e2072.
2. Wiersinga WJ, Currie BJ, Peacock SJ. Melioidosis. *N Engl J Med*. 2012; **367**: 1035–1044.
3. Currie BJ, Fisher DA, Howard DM, Burrow JN, Lo D, Selva-Nayagam S. Endemic melioidosis in tropical northern Australia: a 10-year prospective study and review of the literature. *Clin Infect Dis* 2000; **31**: 981–986.
4. White NJ, Dance DA, Chaowagul W, Wattanagoon Y, Wuthiekanun V, Pitakwatchara N. Halving of mortality of severe melioidosis by ceftazidime. *Lancet* 1989; **2**: 697–701.
5. Goel A, Bansal R, Sharma S, Singhal S, Kumar A Chronic melioidosis presenting with multiple abscesses. *Oxf Med Case Reports.* 2016; 6: 113–116.
